RETRACTED

# Pre-treatment levels of circulating free IGF-1 identify NSCLC patients who derive clinical benefit from figitumumab

**DOI:** 10.1038/sj.bjc.6605972

**Published:** 2010-11-23

**Authors:** A Gualberto, M L Hixon, D D Karp, D Li, S Green, M Dolled-Filhart, L G Paz-Ares, S Novello, J Blakely, C J Langer, M N Pollak

**Affiliations:** 1 The Department of Clinical Development and Medical Affairs, Pfizer Oncology, New London, CT 06320, USA; 2 Department of Pathology and Laboratory Medicine, Warren Alpert Medical School at Brown University, Providence, RI 02903, USA; 3 Department of Thoracic Oncology, MD Anderson Cancer Center, Houston, TX 77030, USA; 4 HistoRx Inc., New Haven, CT 06511, USA; 5 Department of Medical Oncology, Virgen del Rocio University Hospital, Seville 41013, Spain; 6 Department of Medical Oncology, University of Turin, Orbassano, Turin 10043, Italy; 7 Department of Medical Oncology, West Clinic, Memphis, TN 38120, USA; 8 Hematology/Oncology Division, Abramson Cancer Center, University of Pennsylvania, Philadelphia, PA 19104, USA; 9 Department of Medical Oncology, McGill University, Montreal, Quebec H3T 1E2, Canada

**Keywords:** IGF-IR, IGF-1, figitumumab, NSCLC

## Abstract

**Background:**

Phase III trials of the anti-insulin-like growth factor type 1 receptor (IGF-IR) antibody figitumumab (F) in unselected non-small-cell lung cancer (NSCLC) patients were recently discontinued owing to futility. Here, we investigated a role of free IGF-1 (fIGF-1) as a potential predictive biomarker of clinical benefit from F treatment.

**Materials and method:**

Pre-treatment circulating levels of fIGF-1 were tested in 110 advanced NSCLC patients enrolled in a phase II study of paclitaxel and carboplatin given alone (PC) or in combination with F at doses of 10 or 20 mg kg^−1^ (PCF10, PCF20).

**Results:**

Cox proportional hazards model interactions were between 2.5 and 3.5 for fIGF-1 criteria in the 0.5–0.9 ng ml^−1^ range. Patients above each criterion had a substantial improvement in progression-free survival on PCF20 related to PC alone. Free IGF-1 correlated inversely with IGF binding protein 1 (IGFBP-1, *ρ*=−0.295, *P*=0.005), and the pre-treatment ratio of insulin to IGFBP-1 was also predictive of F clinical benefit. In addition, fIGF-1 levels correlated with tumour vimentin expression (*ρ*=0.594, *P*=0.021) and inversely with E-cadherin (*ρ*=–0.389, *P*=0.152), suggesting a role for fIGF-1 in tumour de-differentiation.

**Conclusion:**

Free IGF-1 may contribute to the identification of a subset of NSCLC patients who benefit from F therapy.

The insulin growth factor (IGF) system is comprised of the IGF ligands (IGF-1 and IGF-2), the IGF binding proteins (IGFBPs 1–7) that regulate ligand bioactivity, the cell surface receptors insulin-like growth factor type 1 receptor (IGF-IR) and IGF-2R, the adaptor proteins insulin receptor substrate (IRS)-1 and -2 and downstream signalling pathways (Pollak, 2008). Signalling through the IGF-IR plays important roles in normal growth and development as well as in the initiation and progression of neoplasia (Chitnis *et al*, 2008). There is considerable current interest in targeting the IGF-1 receptor as a therapeutic strategy in oncology, with more than a dozen drug candidates undergoing clinical evaluation (Gualberto and Pollak, 2009). In NSCLC, the IGF-IR has been shown to be frequently expressed in tumour tissue as well as to mediate the proliferation of lung cancer cell lines (Favoni *et al*, 1994). Also, high IGF-1 levels have been associated with higher incidence and aggressiveness of NSCLC (Spitz *et al*, 2002). These data suggest that targeting the IGF-IR could be a viable approach for the treatment of NSCLC.

RETRACTED

Figitumumab (F) is a selective inhibitor of the IGF-IR that has been well tolerated in initial studies (Gualberto, 2010). Figitumumab enhances the tumour growth inhibition of chemotherapy and targeted agents in pre-clinical models (Cohen *et al*, 2005). A recently completed phase II study concluded that F increases the response rate and progression-free survival (PFS) benefit of paclitaxel and carboplatin as first-line treatment of patients with advanced NSCLC (Karp *et al*, 2009). However, pivotal trials of this agent in NSCLC were recently discontinued owing to futility. These results stress the need to identify patient subpopulations that may preferentially benefit from F therapy. This paper summarises a series of preliminary ancillary studies conducted to characterise plasma markers that could identify a subset of patients who derive benefit from the addition of F to standard NSCLC therapy.

## Materials and methods

### Patients

Study 1002 was a multiple-centre, open-label, randomised phase II trial that investigated the efficacy of the combination of F with paclitaxel (P) and carboplatin (C) as treatment for patients with chemotherapy-naïve stage IIIB or IV NSCLC (Karp *et al*, 2009). Briefly, patients had histologically or cytologically confirmed NSCLC not amenable to curative treatment. Eligible patients had at least one unidimensionally measurable lesion according to the Response Evaluation Criteria in Solid Tumours and Eastern Cooperative Oncology Group performance status of 0/1. Eligible patients were randomised 2:1 (PCF arm : PC arm) to receive P at 200 mg m^−2^ intravenously (i.v.) over 3 h and C with area under the plasma concentration–time curve of 6, i.v. over 15–60 min every 3 weeks with or without F at doses of 10 or 20 mg kg^−1^ in two sequential cohorts (PCF10, PCF20). The protocol was conducted in accordance with Good Clinical Practice guidelines and was approved by each participating institutional ethics review boards. All patients signed written informed consent before enrolment.

RETRACTED

### Laboratory assessments

Plasma samples were collected from fasted patients before trial treatments. Levels of total IGF-1, free IGF-1 (fIGF-1), IGF-2, IGFBP-1, IGFBP-2, IGFBP-3, insulin and cotinine were determined at a central laboratory (Department of Pathology and Laboratory Medicine, Brown University, Providence, RI, USA), using the ELISA method. Antibodies and reagents were from Beckman-Coulter Diagnostic System Laboratories (Webster, TX, USA) as follows: total IGF-1 (DSL 10-2800), fIGF-1 (DSL 10-9410), IGF-2 (DSL 10-2600), IGFBP-1 (DSL 10-7810), IGFBP-2 (DLS 10-7100), IGFBP-3 (DSL 10-6600) and insulin (DSL 10-1610). Cotinine was determined using a kit (CO096A) from Calbiotech (Spring Valley, CA, USA). Glucose and creatinine were determined at the local clinical study sites using standard techniques. E-cadherin and vimentin were quantified using fluorescent immunohistochemistry (F-IHC) and an automated analysis system. Briefly, tumour tissues were deparaffinised, hydrated in water and antigen retrieval performed using standard techniques. Incubation with primary antibodies was conducted for 1 h at room temperature. Primary antibodies were mouse anti-E-cadherin (M3612, clone NCH38, 2 *μ*g ml^−1^; Dako, Carpinteria, CA, USA) and mouse anti-vimentin (MS-129, 0.07 *μ*g ml^−1^; Thermo Scientific, Rockford, IL, USA). Each primary antibody was included in a cocktail with rabbit anti-pan-cytokeratin (Z0622, 1:200; Dako) for the identification of epithelial regions and non-nuclear regions. Image capture, review, validation and scoring were carried out using a PM2000 epi-fluorescence microscopy system and AQUAnalysis software (HistoRx, New Haven, CT, USA).

### Statistical analysis

Progression-free survival curves were constructed using the Kaplan–Meier method, and differences analysed by the log-rank test using the MedCalc software (Mariakerke, Belgium). Receiver-operating characteristic (ROC) analysis, area under the curve estimates and significance tests were accomplished using the built-in functions of MedCalc. Cox proportional hazards regression analysis was used to determine biomarker interactions. Biomarker data were analysed using ANOVA and correlations determined using Pearson's correlation tests.

## Results

Pre-treatment plasma fIGF-1 levels identify NSCLC patients who may benefit from the addition of F to standard chemotherapy.

RETRACTED

A total of 156 patients were randomised 2 : 1 to receive PC with or without F at doses of 10 or 20 mg kg^−1^ (PC, PCF10, PCF20). Plasma samples were obtained on cycle 1 day 1 before dosing from 110 of these patients. Patients were 68% men and had a median age of 64 years (range: 36–85). Forty-nine percent of them had tumours of adenocarcinoma histology and 80% were stage IV. Thirty-five patients received PC, 40 PCF10 and 35 PCF20. The overall efficacy results of this trial have been reported previously (Karp *et al*, 2009). Patients receiving the PCF20 regimen had a clinical benefit in terms of PFS of approximately 6 weeks over PC alone, while no clinical benefit over that of PC alone was observed with PCF10 (3.53, 3.60, 5.0 months median PFS for PC, PCF10 and PCF20, respectively, *P*=0.015). Median concentrations of baseline total IGF-1, free IGF-I, total IGF-2, insulin, and IGFBP-1, -2, -3 were, respectively, 219.3, 0.6, 578.1, 23.6, 15.1, 2.3 and 3627.8 ng ml^−1^. Potential biomarker associations with patient demographics were investigated. Higher baseline levels of fIGF-1 were observed in female patients (0.78 ng ml^−1^, 0.22–1.38 95% CI, *N*=36) than in male patients (0.52 ng ml^−1^, 0.07–1.50 95% CI, *N*=74, *P*=0.005), and in patients with tumours of adenocarcinoma histology (0.76 ng ml^−1^, 0.13–1.68 95% CI, *N*=53) than in those with other histologies (0.55 ng ml^−1^, 0.06–1.4 95% CI, *P*=0.03). No other differences were identified.

Progression-free survival was estimated in the subset of patients providing biomarker samples using the Kaplan–Meier method. Median PFS was similar to that in the overall trial population: 2.97, 3.63 and 5.6 months, respectively, for the PC, PCF10 and PCF20 cohorts (*P*=0.002). The ability of pre-treatment biomarker tests to identify patients who experienced prolonged clinical benefit on PCF treatment, for example, PFS longer than 6 months, was investigated using ROC analysis. Receiver operating characteristic curves plot the true positive rate (sensitivity) in function of the false positive rate (100-specificity, if expressed as percentage) at different biomarker cutoff points, and the 95% CI of the value for the area under the ROC curve (AUC) can be employed to test for predictive value (ROC curve AUC must be >0.5 for the test to be potentially useful) (Zweig and Campbell, 1993). Receiver operating characteristic plots were also employed to screen for markers able to identify patients with reduced clinical benefit, for example, patients with PFS shorter than 3 months. Table 1 summarises the AUC values and significance of the ROC analyses for the baseline analytes of patients receiving PCF20. As expected, the AUC 95% CI were wide owing to the small sample size (*N*=35); however, it was observed that high pre-treatment levels of fIGF-1 (at least 0.54 ng ml^−1^) in patients receiving PCF20 were associated (*P*=0.007) with PFS >6 months, whereas low pre-treatment fIGF-1 levels were associated (*P*=0.026) with PFS <3 months. When patients receiving PCF10 and PCF20 were analysed together (*N*=75), significant AUCs (P⩽0.05) were also identified. Figure 1 shows the ROC plots for all patients treated with F (10, 20 mg kg^−1^) using PFS benefit beyond 3, 4, 5 and 6 months as end points. Although our sample size was insufficient to investigate differences in AUC, the results represented in the figure were suggestive that fIGF-1 is a better predictor of long-term clinical benefit of F combination therapy. In contrast, pre-treatment fIGF-1 levels were not predictive of PFS in patients receiving PC only (not shown), suggesting that this parameter was not a general prognostic marker for the outcome of chemotherapy. Of interest, high pre-treatment levels of IGFBP-1 were associated (*P*=0.04) with PFS <3 months (Table 1).

RETRACTED

The potential interaction between pre-treatment fIGF-1 criteria and the PFS benefit derived from F treatment was then investigated using the Cox proportional hazards models. Free IGF-1 cutoff criteria from 0.1 to 0.9 ng ml^−1^ were examined. Useful criteria were found in the range of 0.5–0.9 ng ml^−1^. For PCF20 *vs* PC, the estimated treatment–biomarker interaction terms from Cox proportional hazards models were between 2.5 and 3.5 for fIGF-1 criteria in the 0.5–0.9 ng ml^−1^ range, with one-sided *P*-values of 0.11 (0.5 ng ml^−1^ criterion), 0.09 (0.6 ng ml^−1^ criterion), 0.030 (0.7 ng ml^−1^ criterion), 0.033 (0.8 ng ml^−1^ criterion) and 0.026 (0.9 ng ml^−1^ criterion) adjusted for multiple testing. Hazard ratios for patients with fIGF-1 values above or below the 0.5–0.9 ng ml^−1^ criteria are shown in Figure 2A. Patients above each criterion had a substantial observed improvement in PFS on the PCF20 arm, while only a modest effect was observed below the criterion. For example, the PFS hazard ratio (PCF20/PC) was 4.2 for patients with fIGF-1 above 0.8 ng ml^−1^, but only 1.9 for patients with fIGF-1 equal or below 0.8 ng ml^−1^. A significant biomarker/treatment interaction for PCF10 was only observed at the fIGF-1 >0.8 ng ml^−1^ (*P*=0.027) and >0.9 ng ml^−1^ (*P*=0.04) criteria. Figure 3A–C shows specific examples of Kaplan–Meier curves for all patients in the biomarker cohort (Figure 3A; *N*=110), those with a baseline fIGF-1 level equal or lower than 0.7 ng ml^−1^ (Figure 3B; *N*=64) and those with a baseline fIGF-1 level higher than 0.7 ng ml^−1^ (Figure 3B; *N*=46). Median PFS for patients who had a baseline fIGF-1 level above 0.7 ng ml^−1^ were 2.63 (PC), 3.97 (PCF10) and 6.53 months (PCF20), respectively (*P*=0.0007). In contrast, no apparent differences in median PFS between the treatment cohorts were observed in those who had a baseline fIGF-1 level equal or below 0.7 ng ml^−1^. Additional analysis of PFS by fIGF-1 quartiles further indicated that clinical benefit of F combination therapy increased with baseline fIGF-1 levels. Tumours in patients with plasma fIGF-1 levels at the highest quartile (4th quartile, fIGF-1 ⩾1 ng ml^−1^) derived particular benefit from the addition of F to standard chemotherapy (Figure 4).

RETRACTED

### Effect of the insulin to IGFBP-1 ratio

The findings described above prompted us to investigate the mechanisms underlying the heterogeneity of fIGF-1 levels among NSCLC patients. It is well known that the bioactivity of IGF-1 and IGF-2 is modulated by 6, potentially 7, binding proteins (IGFBPs), of which IGFBP-1 and -3 are the best characterised (Pollak, 2008). Using the Pearson’s parametric correlation test, a significant inverse correlation was identified between pre-treatment fIGF-1 and IGFBP-1 levels (*ρ*=−0.295, *P*=0.005), but no significant association was observed between fIGF-1 and IGFBP-2 (*P*=0.37) or IGFBP-3 (*P*=0.9). Receiver operating characteristic plots were conducted to investigate potential associations between PFS rate and the pre-treatment ratios of IGF-1, IGF-2 and insulin to IGFBP-1, -2 and -3. A high baseline ratio of insulin (*μ*U ml^−1^) to IGFBP-1 (ng ml^−1^) was found to be predictive (*P*=0.05–0.1) of the PFS rate of patients receiving PCF20 at multiple time points in the 3–8 months post-treatment period. No other significant associations were identified.

Insulin/IGFBP-1 ratio cutoffs criteria of 0.6–1 were then examined using Cox proportional hazards models. For PCF20, all cutoff criteria appeared to be potentially useful, with one-sided *P*-values for treatment–biomarker interaction of 0.07 (insulin/IGFBP-1 ratio of 0.5), 0.06 (ratio of 0.6), 0.02 (ratio of 0.7), 0.02 (ratio of 0.8), 0.03 (ratio of 0.9), 0.01 (ratio of 1) and 0.08 (ratio of 1.1), respectively, adjusted for multiple testing (Figure 2B). For PCF10, cutoff criteria of interest were 0.9 (*P*=0.04) and 1 (*P*=0.05). Kaplan–Meier estimates of median PFS in patients enrolled in Study 1002 who had a baseline insulin/IGFBP-1 ratio above 0.8 were 2.83 (PC), 3.86 (PC10) and 5.60 months (PC20), respectively (*P*=0.016; Figure 2D–F).

### Other potential predictors

Other potential predictors of F activity were investigated. These included creatinine and creatine clearance, body mass index, fasting glucose to insulin ratio, the homeostatic model assessment of insulin sensitivity (HOMA) and the quantitative insulin sensitivity check index (QUICKI). None of these parameters reached significance in both the ROC and the Cox biomarker interaction analyses. A potential interaction with smoking was investigated using patient reported smoking habits and measuring pre-treatment cotinine levels, a serum metabolite of nicotine. Cotinine was detected in 0 of 13 patients who declared to have never smoke, eight of 61 patients who declared to be ex-smokers and 12 of 17 smokers. No effect of cotinine levels or smoking status on the PFS of patients receiving F was identified.

RETRACTED

### High plasma fIGF-1 is associated with high vimentin and low E-cadherin expression in NSCLC

We have previously shown that the IGF-IR and other molecules associated to the IGF-IR pathway (e.g. IGF-2R, IRS-1, -2) are overexpressed in NSCLC tumours undergoing epithelial-to-mesenchymal transition (EMT) (Gualberto *et al*, 2009). Epithelial-to-mesenchymal transition is a key feature of tumour infiltration and metastasis that is characterised at a molecular level by the expression of mesenchymal markers, such as vimentin, and the downregulation of epithelial differentiation markers, such as E-cadherin (Kalluri and Weinberg, 2009). We hypothesised that high circulating levels of fIGF-1 could be associated with high IGF bioactivity in the tumour microenvironment, and this could favour EMT. As a first step investigating the relationship between fIGF-1 in plasma and tumour EMT, E-cadherin and vimentin levels were quantified using F-IHC in tumour biopsies of 45 patients enrolled in Study 1002. The relationship between circulating fIGF-1 and tissue marker expression (F-IHC AQUA scores) was investigated using Pearson's correlation analysis. Free IGF-1 correlated directly with tumour vimentin (*ρ*=0.594; *P*=0.021), and inversely with E-cadherin expression (*ρ*=−0.389; *P*=0.152) and the tumour E-cadherin/vimentin ratio (*ρ*=−524, *P*=0.007). Of note, tumours in patients who had high levels of circulating fIGF-1 had barely detectable levels of E-cadherin (Figure 5), suggesting high degree of tissue de-differentiation.

## Discussion

Many targeted therapies are active only for a subset of patients, and the characterisation of predictive biomarkers to identify those patients who are likely to benefit has been a key aspect of drug development. Examples include predicting benefit from trastuzumab therapy in breast cancer by assessing *HER2/neu* amplification (Sauter *et al*, 2009) and from cetuximab in colorectal cancer by assessing *K-ras* mutations (Siena *et al*, 2009). To date, predictive biomarkers for targeted therapies in NSCLC have been defined largely in the context of agents that target the EGF receptor family (Shepherd and Tsao, 2010), although recent data suggest a predictive value of *EML4-ALK* gene fusion for the clinical benefit derived from ALK inhibition (Koivunen *et al*, 2008). We undertook the current investigation to identify potential biomarkers that would allow for the prospective selection of patients who could benefit from the addition of F to standard chemotherapy of NSCLC.

RETRACTED

Higher pre-treatment fIGF-1 levels were found to be predictive of the clinical benefit derived from the addition of F to chemotherapy in NSCLC patients. Although these results require confirmation in larger studies, it is of interest that consistent with our results, preliminary data from a recently discontinued phase III of PCF20 *vs* PC in patients with non-adenocarcinoma NSCLC revealed a biomarker/treatment interaction for baseline levels of fIGF-1. Median overall survival times were 10.2 and 7.0 months, respectively, for patients with a baseline fIGF1 >1 ng ml^−1^ receiving PCF20 and PC alone (Jassem *et al*, 2010). Analysis of this phase III study continues and final results will be discussed elsewhere.

In view of the considerable interindividual heterogeneity in levels of IGFs and their binding proteins, we hypothesise that plasma hormone levels might have particular utility in personalised therapy. This is a departure from the more common paradigm of emphasising molecular characteristics of the tumour in searching for predictive biomarkers. The reasoning underlying this hypothesis is that tumours that develop in a patient with high IGF bioactivity are more likely to become dependent on (or even ‘addicted’ to) IGF-1 receptor signalling, and therefore may be more sensitive to F therapy. Our results suggest that pre-treatment levels of fIGF-1 are predictive of the clinical benefit of F therapy in NSCLC, independent of any tumour characteristics. The possibility that more precise identification of patients who may benefit from IGF-IR targeting could be achieved by the use of algorithms that combines patient hormone levels and tumour characteristics remains open, but could not be explored in this study owing to small sample size. We observed however that tumours of patients with elevated circulating fIGF-1 expressed higher levels of vimentin and lower levels of E-cadherin, suggesting EMT. We speculate that this tumour characteristic is secondary to the hormonal environment. It has been shown previously that IGFs can induce neo-expression of mesenchymal markers and E-cadherin downregulation (reviewed by Julien-Grille *et al* (2005)). Insulin growth factors have also been shown to enhance the phosphorylation of *β*-catenin, causing its dissociation from membrane E-cadherin and translocation to the cytoplasm/nucleus (Playford *et al*, 2000; Morali *et al*, 2001). These interactions are thought to facilitate the coupling of IGF-IR activation with migration, invasiveness and metastasis.

RETRACTED

High insulin to IGFBP-1 ratio was also predictive of the clinical benefit derived from F therapy, and an inverse correlation was observed between fIGF-1 and IGFBP-1. A role for IGFBP-1 in the control of IGF-1 bioactivity has been described previously (Bereket *et al*, 1996; Attia *et al*, 1999). Of note, over 90% of serum IGF-1 circulates in a complex with IGFBP-3 and another glycoprotein, acid-labile subunit (ALS). This complex is large (150 kDa), unable to transverse the endothelial barrier and has a long half-life, acting as a serum reservoir of IGF-1 (Kelley *et al*, 1996). In contrast, IGF-1 bound to IGFBP-1 does not form complexes with ALS, is able to cross the endothelial barrier and is, consequently, more likely to play a role in the regulation of IGF-1 bioactivity at extravascular tissues (Lee *et al*, 1993).

Insulin growth factor binding protein-1 levels and its IGF-1 binding capacity are tightly regulated by insulin, with IGFBP-1, as a result, acting as a bridging molecule between the insulin and IGF systems (Sakai *et al*, 2001; Borai *et al*, 2007). Thus, our data suggest that insulin may affect the risk/benefit of anti-IGF-IR therapy by regulating fIGF-1 levels. This is not in contradiction with other potential effects of insulin on cancer therapy; for example, those mediated by insulin receptors on tumour cells (Gualberto and Pollak, 2009). A role for IGFBP-1 in cancer has not been extensively studied, but it is known that low IGFBP-1 levels are associated with poor prognosis in at least one tumour type, colorectal cancer (Wolpin *et al*, 2009). Further research on IGFBP-1 functions could contribute to a better understanding of the effects of carbohydrate metabolism on cancer outcome. Overall, our data are consistent with previous reports associating low IGF-1 bioactivity with longer overall, disease-free and event-free survival in NSCLC (Chang *et al*, 2002; Han *et al*, 2006). In principle, the utilisation of circulating factors as predictive biomarkers would appear to be more convenient than measurements requiring fresh or frozen neoplastic tissue. However, it should be noted that current assay methodologies, particularly those measuring IGF-1 bioactivity, are controversial and imperfect (Frystyk, 2007). For example, in some applications, measurement of fIGF-1 offers no additional information beyond that provided by total IGF-1 (Juul *et al*, 1997), a measurement which is much more widely used than fIGF-1, but that is itself challenging (Brugts *et al*, 2008a). This issue is further complicated by the relatively small fraction of total IGF-1 bound to IGFBP-1 (Attia *et al*, 1999). In our hands, the fIGF-1 assay had an intra-assay imprecision of approximately 10% at the criteria of interest (0.5–0.9 ng ml^−1^); however, differences were observed across reagent lots. Thus, further analytical validation would be desirable before the prospective use of this assay in randomised studies. Structural studies have recently shown that the binding residues for IGFBP-1 and -3 on IGF-1 are overlapping but distinct (Dubaquié and Lowman 1999; Dubaquié *et al*, 2001). These differences could be exploited to develop new assays for the quantification of the fIGF-1 fraction specifically released from IGFBP-1. Development of such reagents could be important for a more personalised use of anti-IGF-IR therapy.

RETRACTED

This exploratory study was not sufficiently powered for subset safety analysis. No major differences in the frequency or severity of adverse events between subgroups of patients with low *vs* high baseline fIGF-1 were apparent (not shown). Low levels of IGF-1 bioactivity have been associated with increased risk of cardiovascular mortality, whereas fasting IGFBP-1 levels were associated with more favourable cardiovascular risk profiles (Janssen *et al*, 1998; Brugts *et al*, 2008b). Of note, IGF-1 bioactivity changes during the progression of the metabolic syndrome, increasing in parallel to HOMA-IR and hyperinsulinaemia, but decreasing drastically when patients reach frank diabetes (Brugts *et al*, 2010). Insulin growth factor-1 bioactivity is also limited at low total IGF-1 levels (Brugts *et al*, 2010). Thus, treatment with anti-IGF-IR therapy in patients with low levels of total IGF-1 and/or glucose intolerance should be approached with caution. The ongoing analysis of the safety profile of larger F studies may contribute to a better understanding of the potential role of fIGF-1 in the assessment of the risk/benefit of anti-IGF-IR therapy.

In conclusion, our data provide preliminary evidence that fIGF-1 is a predictive biomarker of the clinical benefit, in terms of PFS, of F therapy in NSCLC. Confirmation of these findings in larger studies is needed. We also recognise the need to optimise assay methods and to further study the interactions between serum markers and tumour characteristics in NSCLC and other cancer types in which IGF-IR targeting is currently being investigated.

## Figures and Tables

**Figure 1:** Receiver-operating characteristic curves for fIGF-1 as a predictive maker for PFS benefit at 3–6 months in PCF-treated patients (10–20 mg kg^−1^ F).

RETRACTED

**Figure 2:** (**A**) Hazard ratio of Study 1002 patients receiving treatment with PCF (10 or 20 mg kg^−1^) *vs* PC alone according to baseline fIGF-1 levels. (**B**) A hazard ratio of patients receiving treatment with PCF (10 or 20 mg kg^−1^) *vs* PC alone according to baseline insulin to IGFBP-1 ratio.

**Figure 3:** Kaplan–Meier plots of PFS in Study 1002 patients. (**A**) All patients with available baseline fIGF-1 level data (*N*=110). (**B** and **C**) Patients with baseline fIGF-1 ⩽0.7 (**B**, *N*=64) or >0.7 ng ml^−1^ (**C**, *N*=46). (**D**) All patients with available baseline insulin/IGFBP-1 ratio data (*N*=82). (**E** and **F**) Patients with baseline insulin/IGFBP-1 ratio ⩽0.7 (**E**, *N*=34) or >0.7 ng ml^−1^ (**F**, *N*=48).

**Figure 4:** Progression-free survival of PC, PCF10 and PCF20 patients by fIGF-1 quartile. The central box represents the values from the lower to upper quartile (25–75 percentile). In the box plots, the middle line represents the median. A line extends from the minimum to the maximum value, excluding ‘outside’ values that are displayed as separate points. An outside value is defined as a value that is smaller than the lower quartile minus 1.5 times the interquartile range, or larger than the upper quartile plus 1.5 times the interquartile range (inner fences). These values are plotted with a square marker.

**Figure 5:** Cyanine-5 fluorescence images representative of vimentin and E-cadherin expression in tumours from Study 1002 patients. Insets show cytokeratin (green) and DAPI (blue) fluorescence sample stainings.

**Table 1:** ROC for baseline IGF-IR-related serum analytes in patients receiving PCF20

	**PFS at 3 months**		**PFS at 6 months**	
**Analyte**	**ROC AUC 95% CI**	***P*-value**	**ROC AUC 95% CI**	***P*-value**
Total IGF-1	0.368–0.758	0.566	0.476–0.846	0.140
fIGF-1	0.536–0.852	0.026	0.661–0.933	0.007
IGF-2	0.430–0.811	0.290	0.460–0.834	0.215
Insulin	0.387–0.769	0.457	0.464–0.832	0.213
IGFBP-1	0.531–0.880	0.040	0.405–0.784	0.401
IGFBP-2	0.498–0.862	0.086	0.361–0.752	0.650
IGFBP-3	0.306–0.652	0.842	0.478–0.809	0.178

Abbreviations: AUC=area under the ROC curve; CI=confidence interval; IGF=insulin-like growth factor; fIGF-1=free insulin-like growth factor 1; IGFBP=insulin-like growth factor binding protein; IGF-IR=insulin-like growth factor type 1 receptor; PCF=paclitaxel and carboplatin in combination with figitumumab; PFS=progression-free survival; ROC=receiver operating characteristics.
